# Identification of Hearing Loss-Associated Variants of *PTPRQ*, *MYO15A*, and *SERPINB6* in Pakistani Families

This article has been retracted.

**DOI:** 10.1155/2021/5584788

**Published:** 2021-04-24

**Authors:** Umair Mahmood, Shazia A. Bukhari, Muhammad Ali, Zubair M. Ahmed, Saima Riazuddin

**Affiliations:** ^1^Department of Biochemistry, Government College University, Faisalabad 38000, Pakistan; ^2^Department of Animal Sciences, Quaid Azam University, Islamabad 46000, Pakistan; ^3^Department of Otorhinolaryngology Head and Neck Surgery, University of Maryland School of Medicine, Baltimore, MD 21201, USA

## Abstract

The inner ear is an essential part of a well-developed and well-coordinated hearing system. However, hearing loss can make communication and interaction more difficult. Inherited hearing loss (HL) can occur from pathogenic genetic variants that negatively alter the intricate inner ear sensory mechanism. Recessively inherited forms of HL are highly heterogeneous and account for a majority of prelingual deafness. The current study is designed to investigate genetic causes of HL in three consanguineous Pakistani families. After IRB approval, the clinical history and pure tone audiometric data was obtained for the clinical diagnosis of HL segregating in these three Pakistani families. We performed whole exome sequencing (WES) followed by Sanger sequencing in order to identify and validate the HL-associated pathogenic variants, respectively. The 3-D molecular modeling and the Ramachandran analysis of the identified missense variants were compiled to evaluate the impact of the variants on the encoded proteins. Clinical evaluation revealed prelingual severe to profound sensorineural HL segregating among the affected individuals in all three families. Genetic analysis revealed segregation of several novel variants associated with HL, including a canonical splice-site variant (c.55-2A>G) of *PTPRQ* in family GCFHL-01, a missense variant [c.1079G>A; p.(Arg360Gln)] of *SERPINB6* in family LUHL-01, and an insertion variant (c.10208-10211insCCACCAGGCCCGTGCCTC) within *MYO15A* in family LUHL-011. All the identified variants had very low frequencies in the control databases. The molecular modeling of p.Arg360Gln missense variant also predicted impaired folding of SERPINB6 protein. This study reports the identification of novel disease-causing variants in three known deafness genes and further highlights the genetic heterogeneity of HL in Pakistani population.

## 1. Introduction

A significant portion of our genome, comprised of ~30,000 genes [1, 2], is associated with the development and function of hearing. Pathogenic variants in these genes account for around 50% of hearing loss (HL) cases. Approximately 5% of the world's population is affected with various kinds of HL [3]. HL is the most recurrent sensory disability in humans with a frequency rate of 1–2 : 1000 babies. Worldwide, this targets around 360 million people of different ages [4]. More than 70% of hearing impairments are nonsyndromic with an inheritance of 70-90% autosomal recessive, 10-20% autosomal dominant, and 1-2% X-linked and mitochondrial inheritance [5]. Nonsyndromic recessive hearing loss (NSRHL) genes encode proteins widely spread in different tissues. However, variants in NSRHL genes specifically hinder the intricate inner ear sensory mechanism [6, 7]. For nonsyndromic SNHL, 76 genes have been identified out of the 126 distinct autosomal genetic HL loci [8].

Among populations that have high rates of consanguineous marriages and are isolated based upon geographically, religiously, cultural, and social factors, recessive disorders are found in abundance [9]. In Pakistan, the ratio of consanguineous marriages is extremely high. Because of this, congenital severe hearing impairment accounts for 70% of the total HL cases in Pakistan [10]. Considering these facts, the present study was designed to determine the previously unknown nucleotide basis that was responsible for hearing damage in three large consanguineous Pakistani families affected with HL.

In the hearing process, several hundreds or even thousands of genes are involved in the proper development and functioning of the inner ear neurosensory epithelia. Diverse genes and their expressed protein families (e.g., solute carrier proteins, gap junction, and motor proteins) play orchestrated roles in the various molecular functions of the inner ear, including neurotransmitter release, maintenance of ionic homeostasis, control of adhesion in hair cells, intracellular transport, and protection of hair cell cytoskeleton. Together, all this makes it possible for us to hear sounds [3].

Over the last two decades, we witnessed rapid identification of genes and their pathogenic variants associated with hearing loss in humans. Studies in inbred families were an especially dominant part of this field. In the current study, whole exome sequencing (WES) was used for the identification of causative genes in large consanguineous Pakistani families with the HL phenotype. The current study reports novel variants of three known deafness genes and further highlights the genetic heterogeneity of HL in the Pakistani population.

## 2. Materials and Methods

### 2.1. Subjects and Clinical Evaluation

The study was compiled following the tenets of the Declaration of Helsinki for human subjects, and all the procedures that were followed were preapproved by the Institutional Review Board Committees (HP-00061036) at the University of Maryland School of Medicine, Baltimore, MD, USA, and Government College University, Faisalabad, Pakistan. All the individuals consented in written local combination format for voluntarily inclusion in this project. The families were selected on the basis of (i) inheritance of disease phenotype and (ii) the number of affected individuals (≥3 affected). The family members were interviewed in detail to develop the family pedigree, associated disorders, and their follow-up. The physical examination, medical history, and pure tone audiometry data were assembled to highlight the clinical phenotype.

### 2.2. Whole-Exome Sequencing and Bioinformatics Analyses

WES was used to analyze the variants in the DNA sample of the affected individuals from each family, and the Agilent SureSelect Human Expanded All Exon V5 kit was used to recover genomic libraries and sequenced with an average of 100x coverage on an Illumina HiSeq4000 (Illumina, San Diego, CA, USA). Reads were aligned with the Illumina Chastity Filter with the Burrows-Wheeler Aligner [11]. The GATK UnifiedUnityper module was used to call the variant sites, and the variant quality score recalibration method was used to filter single nucleotide variants [12]. The filtration of candidate variants, DNA sequencing, and PCR amplification was also performed [13]. Primer 3 (http://bioinfo.ut.ee/primer3-0.4.0/) was used to design the primers used for PCR.

### 2.3. Molecular Modeling

The three-dimensional (3-D) structures of wild-type and mutant proteins SERPINB6 were generated by Phyre2 (http://www.sbg.bio.ic.ac.uk/phyre2/html/page.cgi?id=index) by using an intense mode option. The Chimera online tool was used to visualized PDB structure of protein that was subsequentially further analyzed. MolProbity was used to generate Ramachandran plots for both the wild-type and mutant protein PDB structures. Clustal Omega (https://www.ebi.ac.uk/Tools/msa/clustalo/) was used to align the sequence of the closely related species.

## 3. Results

### 3.1. Clinical Data

As part of our ongoing efforts to ascertain and clinically and genetically characterize Pakistani families with hearing loss [14, 15], three new large consanguineous families were enrolled from the Punjab province of Pakistan after approval from the Institutional Review Board (IRB) of University of Maryland School of Medicine, Baltimore, MD, USA, and the Government College University, Faisalabad, Pakistan. In all affected individuals, HL was observed from birth, except for the affected individuals of family GCFHL-01 who had progressive HL and were diagnosed after 4-5 years of age. The audiometric profile of affected members of family LUHL-01 revealed moderate to severe hearing damage, and the affected members of family LUHL-011 showed severe to profound HL. Previous medical history and clinical diagnosis did not reveal any apparent comorbidity with HL. Romberg and Tandem gait tests revealed normal vestibular system in affected individuals of all families. The peripheral vision loss, cornea opacity, or night blindness was not observed during ophthalmoscopic examination in any individuals from the included families.

### 3.2. Mutation Detection and Molecular Modeling

WES of three large consanguineous Pakistani families was performed to analyze the pathogenic variants for NSHL. The novel splicing variant c.55-2A>G of *PTPRQ* was detected as cosegregating in the affected individuals of families GCFHL-01, while an insertion variant c.10208-10211insCCACCAGGCCCGTGCCTC of *MYO15A* segregating with HL was found in family LUHL-011 (Figures 1(a) and 2(a)). Finally, a novel predicted missense variant c.1079G>A (p.(Arg360Gln)) of *SERPINB6* was identified in family LUHL-01 (Figures 1(a) and 2(a)). All the identified variants were predicted pathogenic by various in silico algorithms, were either absent or had low allele frequency in gnomAD database, and were classified as pathogenic or likely pathogenic according to ACMG classification (Table 1). Furthermore, the p.(Arg360Gln) predicted missense variant replaces an evolutionary conserved residue in the encoded protein (Figure 1(c)). All three variants are located in the functional domains of encoded proteins (Figure 2(a)).

### 3.3. Molecular Modeling

To determine the impact of p.Arg360Gln missense variant on the encoded SERPINB6 protein, the 3-D structure of wild-type and mutated proteins were generated using the online bioinformatics tool Phyre2 (http://www.sbg.bio.ic.ac.uk/phyre2/html/page.cgi?id=index) and were visualized through Chimera software. The p.Arg360Gln replacement resulted in a smaller and negatively charged residue (Gln) as compared to the large and positively charged wild-type residue (Arg), which is predicted to cause alterations in the ionic interactions. This accounts for the aberrant interactions with neighboring residue alanine at position 354 (Figure 2(b)) and also might further disturb the secondary protein structure.

We also used the MolProbity tool to generate Ramachandran plots for both wild-type and mutant protein PDB structures. In the Ramachandran plot, the wild SERPINB6 protein shows that 88% of the residues reside within a favorable region and 96% residues are in allowed region, while 14 were outliers. In contrast, for the p.Arg360Gln mutant protein, 68% of the residues are found in the favored region, 86% are found in the allowed region, and 53 were outliers (Figure 2(c)). Overall, there is a significant difference in amino acid distribution of wild type versus mutant type (Figure 2(c)).

## 4. Discussion

Our study further expands the genetic landscape of inherited variants of HL-associated genes in the Pakistani population and revealed three novel variants in three known nonsyndromic deafness genes, *MYO15A, PTPRQ*, and *SERPINB6*. Although variants in *MYO15A* are a commonly known cause of HL worldwide (including the Pakistani population) [16], variants of *PTPRQ* and *SERPINB6* are relatively rare. In fact, to our knowledge, the p.(Arg360Gln) variant found in SERPINB6 is only the fourth ever reported allele that is associated with HL in humans [17, 18]. *SERPINB6* is located on the chromosome at position 6p25.2 and encodes serpin (serine protease inhibitor) superfamily and subfamily ovalbumin-serpin B member 6, cytoplasmic anti-proteinase (CAP) protein. In the inner ear of the mouse, SERPINB6 is highly enriched in the organ of Corti sensory cells; however, expression is also found in the stria vascularis and spiral limbus region [19, 20]. Mice lacking SERPINB6A exhibit progressive degeneration of cochlear sensory cells and HL [19, 20]. We observed moderate to severe HL in family LUHL-01. However, it is not possible to determine if the hearing loss observed is progressive in nature or not, considering we only have data from a single audiometric report. Previous reports in human subjects with SERPINB6 variants also lack the longitudinal analysis of hearing loss phenotype [17, 18]. We plan to follow up the evaluation of hearing phenotype in family LUHL-01 in future after the COVID-19 pandemic restriction lessen.

*PTPRQ*, located at chromosome 21q21.31, encodes the protein tyrosine phosphatase receptor Q (EC 3.1.1.48), a member of the protein tyrosine phosphatase receptor family type III. Previously, variants in *PTPRQ* have been reported for having dominant (DFNA73) [21], as well as recessively inherited (DFNB84) forms of nonsyndromic HL in human [22, 23]. We identified a novel splice variant (c.55-2A>G) of *PTPRQ* inherited in a recessive manner in family GCFHL-01. We did not observe HL among carriers of c.55-2A>G variant in family GCFHL-01. *In silico* analysis revealed cryptic splicing due to c.55-2A>G variants, which is predicted to cause exon skipping and premature truncation of the encoded protein, likely indicating a loss-of-function disease mechanism in the affected individuals of family GCFHL-01.

An inframe insertion variant in the carboxy tail FERM domain (Figure 2(a)) of MYO15A also was observed co-occurring with HL in family LUHL-011. Pathogenic variants of *MYO15A* have been extensively reported in families sensorineural nonsyndromic severe to profound HL [16]. Previously, a different insertion deletion (c. c.10208_10209delAGinsACCAGGCCCGTGCAGCTC) variant at the same nucleotide position, mutated in family LUHL-011, was documented in another large Pakistani family [16], which could be coincidental or a mutation hot spot. In conclusion, our study further expands the genetic landscape of HL-associated variants of known deafness genes and provides information that can improve molecular diagnostics and genetic counseling for families segregating prelingual HL.

## Figures and Tables

**Figure 1:** Family pedigrees, hearing loss (HL) phenotype and causative alleles. (a) Segregation of HL causing alleles in three Pakistani families. Double lines indicate consanguineous families, empty symbols represent unaffected individuals, and filled symbols affected individuals. The genotypes of the identified variants are also shown for each of the participating family members. All families had autosomal recessive mode of inheritance for HL. (b) Audiometric air conduction thresholds from the proband of each Pakistani family revealed varying degree of HL. (c) ClustalW multiple amino acid sequence alignment shows evolutionary conservation of arginine at position 360 of SERPINB6.

**Figure 2:** Protein structure, molecular modeling, and Ramachandran plots. (a) Schematic representations of PTPRQ, SERPINB6, and MYO15A proteins along with HL-causing variants were identified in Pakistani families. (b) 3-dimentional molecular modeling of SERPINB6. Protein secondary structures generated by Phyre2 are shown in respective colors: helix, cyan; strand, purple; and coils, green. The protein surface is displayed in a meshwork. Concerned residue is shown in firebrick color, while the aberrant hydrogen bonding due to p.Arg360Gln variant is displayed in golden yellow color. (c) Ramachandran plots of both wild and mutant protein PDB structures; the wild structure shows 88% of the residues existing in the favored region, and 96% of the residues are located in the allowed region, but 68% of the residues in mutant structure are found in the favored region and 86% are in the allowed region, respectively.

**Table 1:** Genes, identified variants, and their American College of Medical Genetics and Genomics (ACMG) classification.

Family	Gene	cDNA change	Protein change	CADD	GnomAD	Mutation taster	Polyphen2	ACMG classification
GCFHL01	*PTPRQ*	c.55-2A>G	N/A	N/A	N/A	Disease causing	N/A	Pathogenic (PVS1, PM2, PP3, and PP5)
LUHL011	*MYO15A*	c.10208-10211insCCACCAGGCCCGTGCCTC	N/A	N/A	N/A	Disease causing	N/A	Pathogenic (PVS1, PM2, PP3, and PP5)
LUHL-01	*SERPINB6*	c.1079G>A	p.(Arg360Gln)	N/A	0.001	Disease causing	Benign	Likely pathogenic (PS3, PP2, PP3, and BP4)

CADD: Combined Annotation Dependent Depletion (https://cadd.gs.washington.edu/); GnomAD: https://gnomad.broadinstitute.org. PVS1: pathogenic very strong [null variant (nonsense, frameshift, canonical ±1 or 2 splice sites, initiation codon, single, or multiexon deletion) in a gene where LOF is a known mechanism of disease]; PM2: pathogenic moderate 2 [absent from controls (or at extremely low frequency if recessive) in Exome Sequencing Project, 1000 Genomes Project, or Exome Aggregation Consortium]; PP3: pathogenic supporting 3 [multiple lines of computational evidence support a deleterious effect on the gene or gene product (conservation, evolutionary, splicing impact, etc.)]; PP5: pathogenic supporting 5 [reputable source recently reports variant as pathogenic, but the evidence is not available to the laboratory to perform an independent evaluation]; BP4: benign supporting 4 [benign computational verdict because of 1 benign prediction from GERP vs. no pathogenic predictions].

## Data Availability

The data used to support the findings of this study are available from the corresponding author upon request.
